RETRACTED

# A Comparison of Early Rehabilitation in the Intensive Care Units of Patients With Severe COVID-19: A Propensity Score Matching Analysis

**DOI:** 10.7759/cureus.31328

**Published:** 2022-11-10

**Authors:** Kohji Iwai, Yasuyuki Tsujita

**Affiliations:** 1 Division of Physical Therapy, Faculty of Rehabilitation and Care, Seijoh University, Tokai, JPN; 2 Department of Critical and Intensive Care Medicine, Shiga University of Medical Science, Otsu, JPN

**Keywords:** propensity score matching analysis, single-center retrospective study, early rehabilitation, intensive care unit, covid-19

## Abstract

Aim

This study aimed to investigate early rehabilitation in the intensive care unit (ICU) for patients with severe coronavirus disease 2019 (COVID-19) who require mechanical ventilation

Methods

Twenty patients with severe COVID-19 (COVID-19 group) who were admitted to the ICU between April 2020 and March 2022 were included. For the control (non-COVID-19) group, 20 individuals were selected among ICU patients admitted between April 2018 and March 2020. The controls were propensity score-matched by age, sex, and Sequential Organ Failure Assessment (SOFA) score.

Results

In the COVID-19 group, the percentage of extubated patients was significantly higher. Furthermore, mechanical ventilation and lengths of ICU stay were also significantly longer. There were no significant differences in discharge outcomes or mortality, but there was a significant difference in the number of muscle relaxants and steroid treatments utilized with the COVID-19 group, requiring more of these medications. The percentage of patients who achieved sitting on the edge of a bed was also significantly higher in the COVID-19 group, but the days between the first rehabilitation and first sitting were significantly greater in this group.

Conclusion

Early rehabilitation of patients with COVID-19 may be an effective measure to promote recovery. However, continued investigation is warranted.

## Introduction

SARS-CoV-2 infection was first reported in Wuhan, China, in December 2019, and it has since been spreading worldwide. Although most patients with coronavirus disease 2019 (COVID-19) show mild to moderate symptoms, about 5% are admitted to the intensive care unit (ICU) due to respiratory failure and requirements for mechanical ventilation [1]. Pulmonary rehabilitation has proven to be effective for patients who required mechanical ventilation [2]. In addition, there have been many reports, including our retrospective study, on the effects and benefits of early rehabilitation in the ICU when performed by a physical therapist [3-6]. Patients with COVID-19 need rehabilitation programs to deal with the consequences of mechanical ventilation and prolonged inactivity [7,8]. However, whether early rehabilitation in the ICU for patients with severe COVID-19 who require mechanical ventilation is similarly effective compared to that in critically ill patients has not been fully investigated.

RETRACTED

Thus, this study aims to examine the effect of early rehabilitation in the ICU for patients with severe COVID-19 using propensity score matching, with our previously reported data as a control [6].

## Materials and methods

Study design and participants

This retrospective study included patients admitted to the emergency ICU between April 2018 and March 2022 at a single hospital in Japan (Shiga University of Medical Science Hospital). Patients who underwent cardiovascular surgery in the coronary care unit, patients who spent only one night in the ICU, and pediatric patients aged less than 18 years were excluded according to our previous report [6]. A physical therapist was assigned to the ICU starting in April 2018, and critically ill patients admitted to the ICU from April 2018 to March 2020 were designated as the control group (non-COVID-19 group). Our hospital began accepting patients with COVID-19 in April 2020, with the main indication for ICU admission being severe respiratory failure requiring intubation and management. Of the 22 patients with severe COVID-19 admitted to the ICU between April 2020 and March 2022, two were excluded. This was because one patient left the ICU before rehabilitation intervention, and another one remained hospitalized after treatment due to another illness. Hence, the remaining 20 patients were selected as part of the COVID-19 group. Of the 383 patients in the non-COVID-19 group, the 166 who received no rehabilitation intervention were excluded. The remaining 217 underwent propensity score matching by age, sex, and Sequential Organ Failure Assessment (SOFA) score against the 20 patients in the COVID-19 group, and the 20 patients were selected for the non-COVID-19 group (Figure 1).

**Figure 1:** Flowchart of patient selection

This study conformed to the principles of the Declaration of Helsinki and was approved by the Research Ethics Committee of Seijoh University (approval number: 2022C0003). The requirement for written informed consent was waived because all data was anonymized. Informed consent was obtained in the form of opt-out.

Management and rehabilitation of patients

Sedation and analgesia in mechanically ventilated patients were managed according to the guidelines proposed by the Japan Society of Respiratory Care Medicine in the non-COVID-19 group [6] and the COVID-19 group. Additionally, the patients in the COVID-19 group were sedated and placed in a prone position for 48 hours after their admission to the ICU, after which their respiratory condition was closely controlled to avoid excessive inspiratory effort.

RETRACTED

For the non-COVID-19 group, the patients were distributed under the management of various medical departments: six in the emergency department (three cases of sepsis, one case of severe trauma, one case of acute respiratory failure, and one case of acute renal failure), three in the cardiology department (two cases of severe irregularities and one case of heart failure), three in the gastroenterology department (two cases of peritonitis and one case of esophageal cancer), three in the otolaryngology department (one case of thyroid cancer, one case of tongue cancer, and one case of cancer of the nasal cavity), two in the dermatology department (one case of gas gangrene and one case of airway burn), one in the orthopedics department (cervical myelopathy), one in the neurosurgery department (subarachnoid hemorrhage), and one in the respiratory medicine department (acute respiratory failure). All cases from the COVID-19 group were handled by the respiratory medicine department. In both groups, a multidisciplinary team composed of doctors, nurses, registered dietitians, pharmacists, clinical engineers, and physical therapists shared patient information, set basic goals in accordance with the rehabilitation protocol, and implemented early rehabilitation as soon as possible (Figure 2) [6]. The definition of sitting on the edge of a bed was determined by checking for improvement in the state of consciousness with reduced sedation, as well as respiratory and hemodynamic stability. However, patients with COVID-19 were kept in a prone position for 48 hours or longer after ICU admission, depending on their respiratory status. The nurses working in the red zone handled the patients when postural drainage was a priority under sedation. Once both respiratory and circulatory status was stabilized, the physical therapist entered the red zone to initiate early rehabilitation. The first day of rehabilitation was defined as the date the physical therapist began the intervention.

**Figure 2:** Rehabilitation protocol for patients in the intensive care unit in our hospital RASS: Richmond Agitation-Sedation Scale, RR: respiratory rate, SpO2: saturation of percutaneous oxygen, FiO2: fraction of inspiratory oxygen, PEEP: positive end-expiratory pressure, S-G: Swan-Ganz catheter, IABP: intra-aortic balloon pumping, PCPS: percutaneous cardiopulmonary support, HR: heart rate, ECG: electrocardiogram

Early rehabilitation sessions were carried out once a day for 20-60 minutes per session in both groups. During the period of the inclusion of eligible patients, one physical therapist was consistently responsible for the exercise rehabilitation regimens approved by the ICU doctors for all patients [6].

RETRACTED

Data collection

Data collection was performed in accordance with our previous report [6]. Patient data, including sex, height, age, and SOFA score, were recorded at ICU admission in the two groups. The duration of mechanical ventilation and the percentage of patients who underwent extubation and tracheotomy were extracted from medical records. In our hospital, the main indications for tracheotomy were prolonged mechanical ventilation for more than two weeks, patients who were expected to require long-term ventilator management, and completion of reintubation. The lengths of both ICU and hospital stays, as well as outcomes at discharge (discharge to home, transfer, or death), were also noted from the medical records [6]. In addition, medication status (muscle relaxant, steroid treatment, and nitric oxide inhalation therapy) and comorbidities were included in the analysis. The indices of the progress of rehabilitation conformed to our previous reports [6] and included the number of days from ICU admission to the day when the patient first underwent rehabilitation and when the patient first sat. When sitting and standing exercises were performed, the therapist provided bedside assistance, being careful to avoid aspiration, and the amount of assistance provided was adjusted according to the patient’s stability. With both groups receiving rehabilitation intervention, each was surveyed for the percentage of rehabilitation program implementation. However, since it was difficult to introduce rehabilitation equipment in the red zone where the COVID-19 group had entered, the percentages of contracture prevention, sitting, and standing were investigated. In addition, from the standpoint of safety management, the maximum load practice was limited to the standing position, and the walking exercise was not recommended.

Statistical analysis

Normally distributed data are expressed as mean ± standard deviation (SD), while non-normally distributed variables are expressed as medians. For continuous variables, the Wilcoxon signed-rank sum test was applied depending on the validity of the normality assumption. The chi-square test was used to assess categorical variables.

The Statistical Package for the Social Sciences (SPSS) (IBM SPSS Statistics, Armonk, NY, USA) was used for all statistical analyses. The results were considered statistically significant if the two-tailed p-value was less than 0.05.

## Results

A comparison of the basic information of the COVID-19 and non-COVID-19 groups is shown in Table 1. All patients underwent rehabilitation, and extracorporeal membrane oxygenation and assisted circulation devices were not used in either group. No physical therapist was infected, and no adverse effects were recorded. The percentage of patients undergoing continuous hemodiafiltration was significantly higher in the non-COVID-19 group (0% versus 50%, p<0.001). Eighteen patients in the non-COVID-19 group and 20 in the COVID-19 group were managed in the ICU with mechanical ventilation. The percentage of extubation was significantly higher in the COVID-19 group (80% versus 44.4%, p=0.026). In addition, the duration of mechanical ventilation and the length of ICU stay were significantly longer in the COVID-19 group (p=0.008 and p=0.004, respectively). There was no significant difference in the length of hospital stay, discharge outcomes, or mortality between the two groups. In terms of medications used, there was a significant increase in the number of muscle relaxants (10% versus 85.8%, p<0.001) and steroid treatments (20% versus 100%, p<0.001) used in the COVID-19 group. There was no significant difference in comorbidities between the two groups (Table 2). The percentage of patients who achieved sitting on the edge of a bed was also significantly higher in the COVID-19 group (90% versus 45%, p<0.016); however, the days from the first rehabilitation (p<0.001) and first sitting (p=0.001) were significantly greater in the COVID-19 group (Table 3).

RETRACTED

**Table 1:** Baseline characteristics of patients in the non-COVID-19 group and COVID-19 group COVID-19: coronavirus disease 2019, SOFA: Sequential Organ Failure Assessment, ICU: intensive care unit, IQR: interquartile range, stand diff: standardized difference

	Non-COVID-19 group (April 2018-March 2020) (N=20)	COVID-19 group (April 2020-March 2022) (N=20)	p-value	stand diff
Gender, male, n (%)	13 (65)	14 (70)	0.906	0.10
Height, cm	160.8±13.3	166.5±9.5	0.238	0.49
Age, year	64.5±13.3	56.0±15.6	0.083	0.59
SOFA score	8.7±2.9	7.9±2.2	0.607	0.30
Patients on ventilator, n (%)	18 (90)	20 (100)	0.244	0.70
Extubation, n (%)	8 (44.4)	16 (80)	0.026	0.79
Tracheotomy, n (%)	5 (27.8)	4 (20)	0.568	0.18
Duration of ventilation, days	3.6±2.1	8.3±4.7	0.008	1.40
Continuous hemodiafiltration, n (%)	10 (50)	0	<0.001	1.41
Polymyxin B-immobilized fiber column direct hemoperfusion, n (%)	2 (10)	0	0.147	0.47
Length of ICU stay, days (IQR)	6 (3-8)	10.5 (6-15.8)	0.004	0.83
Length of hospital stay, days (IQR)	27 (13.8-59.5)	26.5 (19-39)	0.925	0.28
Discharge to home, n (%)	7 (35)	11 (55)	0.236	0.41
Transfers, n (%)	7 (35)	7 (35)		0.00
Death, n (%)	6 (30)	2 (10)		0.51

**Table 2:** Comparison of treatment and comorbidities COVID-19: coronavirus disease 2019

	Non-COVID-19 group (April 2018-March 2020) (N=20)	COVID-19 group (April 2020-March 2022) (N=20)	p-value
Muscle relaxant, n (%)	2 (10)	17 (85)	<0.001
Steroid treatment, n (%)	4 (20)	20 (100)	<0.001
Nitric oxide inhalation therapy, n (%)	2 (10)	4 (20)	0.331
Pulmonary disease, n (%)	4 (20)	4 (20)	0.653
Cardiac disease, n (%)	6 (30)	5 (25)	0.723
Cancer, n (%)	5 (25)	4 (20)	0.500
Hypertension, n (%)	7 (35)	6 (30)	0.736
Diabetes mellitus, n (%)	5 (25)	2 (10)	0.204
Hyperlipidemia, n (%)	4 (20)	5 (25)	0.500

RETRACTED

**Table 3:** Comparison of rehabilitation program COVID-19: coronavirus disease 2019, IQR: interquartile range

	Non-COVID-19 group (April 2018-March 2020) (N=20)	COVID-19 group (April 2020-March 2022) (N=20)	p-value
Days to first rehabilitation, days (IQR)	1 (1-2)	4.5 (3-7)	<0.001
Prevention of contractures, n (%)	19 (95)	18 (90)	0.500
Sitting on the edge of the bed, n (%)	9 (45)	18 (90)	0.016
Days to first sit, days	2.9±1.5	6.7±4.9	0.001
Standing, n (%)	1 (5)	2 (10)	0.500

## Discussion

The non-COVID-19 group had a lower percentage of extubation (44.4%), with some patients leaving the ICU intubated. Therefore, the duration of ventilation is likely to be biased, while early rehabilitation may have contributed to the higher percentage of extubation in the COVID-19 group. This may also be associated with the significantly higher number of patients in the COVID-19 group who performed sitting on the edge of a bed, which increased lower lung aeration and tidal volume, possibly contributing to the improvement of arterial oxygenation [6]. Since positional management was prioritized over weaning, the length of ICU stays tended to be longer in the COVID-19 group. However, the duration of stay in the ICU of COVID-19 patients in the previous report was 12 days (median), and the duration of mechanical ventilation was 10-11 days (median) [9,10], which is generally similar to those in our hospital.

In general, there were no significant differences in clinical outcomes between the two groups. However, 35% of patients with COVID-19 were transferred to the hospital despite an average age of 56 years. This may be due to the significantly higher number of muscle relaxants and steroid treatments used, as well as the significantly longer duration of mechanical ventilation in the COVID-19 group. A previous report suggested that ICU-acquired weakness (AW) is present in 69% of COVID-19 patients admitted to the ICU [11]. This suggests that protein catabolism is more likely to occur with muscle relaxants, sedatives, steroids, and mechanical ventilation [12]. Moreover, it has been reported that coronaviruses may have detrimental immune-mediated effects on myofibrils [13]. Musheyev et al. [14] suggested that most COVID-19 patients still had significant unresolved medical issues at discharge. Therefore, due to a combination of these factors, it is expected that a notable percentage of patients will take longer to resume daily activities after leaving the ICU.

RETRACTED

The higher percentage of patients who were able to sit on the edge of a bed in the COVID-19 group was probably due to the absence of catheter devices used in blood purification therapy, which, if present, would cause a hindrance to patients attempting to sit on the edge of a bed. Additionally, the patients were in the ICU for a longer period of time, which naturally provided more opportunities for them to sit. It is also possible that there were fewer non-lung organ failures in these patients. Regarding the percentage of patients who achieved the first rehabilitation and then the day of the first sitting, the timeline was significantly longer in the COVID-19 group. This may have been influenced by the unique respiratory and positional management of the COVID-19 group after ICU admission. Rehabilitation intervention should be initiated within 2-4 days of ICU admission [15], which was generally achieved in both groups.

This study has several limitations. Firstly, it was a single-center, retrospective study that included only a small number of patients. This could have affected the age matching and overall matching performed. Multicenter studies are required in the future to obtain more robust results. Secondly, the non-COVID-19 group involved a range of diseases, which may have influenced the clinical outcomes due to the differences in the course of each disease. Thirdly, ICU-AW was not evaluated. To prove the effectiveness of early rehabilitation in the future, it would be necessary to prepare indices for daily activities, such as the functional status score for the ICU, and functional indices, such as the medical research council score.

## Conclusions

In the COVID-19 group, 80% of patients were extubated in the ICU. The duration of mechanical ventilation and ICU stay were significantly longer in the COVID-19 group, but these values were not different from those previously reported. In addition, although 35% of patients with COVID-19 were transferred to a different hospital, the percentage of patients sitting on the edge of a bed was significantly higher. Thus, early rehabilitation of patients with COVID-19 may be an effective measure to promote recovery. However, continued investigation is warranted.
